# Model Test and Numerical Simulation of Water Conservancy Foundation Bearing Capacity

This article has been retracted.

**DOI:** 10.1155/2022/7386178

**Published:** 2022-08-31

**Authors:** Jiajia Li

**Affiliations:** College of Water Conservancy and Hydropower Engineering, Sichuan Agricultural University, Ya'an City, Sichuan Province 625014, China

## Abstract

In order to further improve the construction quality of water conservancy projects under different soil conditions and ensure the safety, stability, and durability of water conservancy project foundation construction under special circumstances, this study takes the bearing capacity of water conservancy land foundation as the research direction, takes frozen soil foundation and bag gravel pier composite foundation as examples, and further optimizes the parameters of foundation bearing capacity by using the theory of foundation ultimate bearing capacity and related algorithms. The P-S curve of bearing capacity shows that when the foundation is frozen to −15°C and the foundation sum is about 190 kN, the P-S curve trend at this time changes significantly, which is not different from the indoor simulation result of 170 kN. The final numerical analysis of foundation bearing capacity is relatively reliable, which can provide a powerful reference for the calculation of foundation bearing capacity of hydraulic engineering.

## 1. Introduction

In recent years, with the rapid development of the construction industry, all kinds of construction projects have emerged endlessly, and the expansion of the project scale also puts forward higher requirements for the foundation of construction projects. On the one hand, under the existing circumstances, there are less and less site soils that can be directly treated with natural foundation, so more and more buildings are built on special soil such as soft soil. On the other hand, with the continuous expansion of the building scale, the self-weight, floor height, and load of the building also increase, and the existing buildings have higher and higher requirements for the bearing capacity of the foundation [1]. Generally, composite foundation treatment is adopted in construction projects, and other foundations such as the same pile foundation have obvious advantages. However, for the foundation engineering in some special areas, such as frozen soil area, as well as bag gravel pier composite foundation treatment, we must pay attention to the foundation bearing capacity experiment, as shown in Figure 1. Through the foundation bearing capacity model test to simulate the in situ load test on the construction site, ensure the reliable bearing capacity data of the construction, and ensure the safety and durability of the foundation construction of water conservancy projects.

## 2. Literature Review

Ti and others regard geosynthetics as a material to increase the strength of soil, which is one of the materials used in civil construction. There are many kinds of geosynthetics, which usually use high molecular polymers as raw materials, including synthetic fibers, geogrids, geotextiles, synthetic rubber, and composite geosynthetics, and apply them to projects to improve the bearing capacity and deformation capacity of soil [2]. Zhang et al. believe that geosynthetics are a new engineering material with great vitality. They study geosynthetics, summarize the development of geosynthetics, and make statistics on the classification of geosynthetics. Geosynthetics are classified into four categories, namely, geomembrane, geotextile, geotextile composite, and geotechnical special materials, and their functions and application scope are classified and integrated, which can be divided into six types: reinforcement, drainage, seepage prevention, filtration, isolation, and protection [3]. Obaidat et al.'s research on adding geosynthetics to urban asphalt pavement found that, since the 1970s, the asphalt used in the pavement has been seriously scarce. Therefore, the pavement constructed in the early stage is thin and of poor quality. In the later stage, they face a large number of repair and rectification projects, which not only increases the amount of work but also is a major problem in terms of funds. In the later construction, they applied geosynthetics to subgrade treatment. Through reasonable design and construction, they greatly improved the subgrade bearing capacity, improved the seismic performance of the subgrade, and improved the service life of the pavement, which has great technical and economic value. Geotextile can withstand high temperature of 170°C. It has very large deformation characteristics, which can effectively limit the generation and development of cracks [4]. In addition, Yin et al. also studied the repair and reconstruction of the old pavement, combined with the construction of geosynthetics, paved the middle crack prevention layer, made full use of the reinforcement, isolation, drainage, and filtration functions of geotextiles, extended the service life of the road, and maintained and repaired the existing urban roads more economically [5]. In their research on the application and construction of geosynthetics in hydraulic engineering, Ren et al. found that impervious geosynthetics are often damaged by stones or other sharp objects, and the membrane will also be damaged by the jacking force of gas or liquid. In addition, temperature, humidity, gravity, and so forth will damage impervious geosynthetics. They are a new geotechnical engineering material made of synthetic fiber, plastic, and glass fiber as raw materials. In recent years, it has been widely used in water conservancy projects, mainly in water conservancy seepage prevention projects [2].

## 3. Finite Element Simulation of Ultimate Bearing Capacity of Engineering Foundation

### 3.1. Basic Theory of Ultimate Bearing Capacity of Foundation

#### 3.1.1. Limit Equilibrium Method

Limit equilibrium method is the most widely used stability analysis method in geotechnical engineering. It is used to calculate an equilibrium relationship between the external force borne by the soil and its internal strength near the limit state and can analyze the stability of the soil [6]. The calculation formula is as follows:

(1) $$\begin{array}{c} \left\{\begin{array}{c} p_{k}=cN_{c}+\gamma DN_{q},\\ N_{c}=\left[{\text{tan}}^{4}\left(45^{\circ }+\frac{\phi }{2}-1\right)\cot\phi \right],\\ N_{q}={\text{tan}}^{4}\left(45^{\circ }+\frac{\phi }{2}\right). \end{array}\right. \end{array}$$

It is assumed that the foundation ground is rough and uneven, and the influence of soil bulk density and overlying earth pressure is considered. When the soil mass in the foundation is subject to overall shear failure, forming a sliding surface up to the base, the soil part under the base will slide with the foundation, and this process will form an elastic equilibrium state [7]. The calculation formula in this case is as follows:

(2) $$\begin{array}{c} \left\{\begin{array}{c} p_{k}=cN_{c}+\gamma DN_{q}+\frac{1}{2}\gamma BN_{\gamma },\\ N_{c}=\left(N_{q}-1\right)\cot\gamma ,\\ N_{q}=\frac{\exp\left[\left(3\pi /2-\phi \right)\tan\phi \right]}{2{\text{cos}}^{2}\left(45^{\circ }+\phi /2\phi /2\right)},\\ N_{\gamma }=1.8\left(N_{q}-1\right)\tan\phi . \end{array}\right. \end{array}$$

After that, Meyerhof also considered the influence of the shear strength of the soil above the bottom of the foundation. He believes that the ultimate bearing capacity of the foundation is composed of four parts; that is, the force caused by the side friction of the foundation is increased, so he puts forward the following formula:

(3) $$\begin{array}{c} P_{k}=cN_{c}+qN_{q}+\frac{1}{2}\gamma BN_{\gamma }+\frac{2fD}{B}. \end{array}$$

Hansen proposed that the calculation of bearing capacity should consider the effects of different foundation shapes, the degree of load inclination and eccentricity, and the buried depth of the foundation. The empirical coefficient is used to modify the foundation bearing capacity coefficient, and the following formula is proposed:

(4) $$\begin{array}{c} P_{k}=cN_{c}s_{c}d_{c}i_{c}+qN_{q}s_{q}d_{q}i_{q}+\frac{1}{2}\gamma BN_{\gamma }s_{\gamma }d_{\gamma }i_{\gamma }. \end{array}$$

#### 3.1.2. Slip Line Method

The slip line method divides the soil into two parts, plastic zone and rigid zone. According to the stress yield condition, equilibrium equation, and stress boundary condition, the different distributions of stress, displacement, and velocity in the plastic zone can be solved, and the boundary stress within the foundation can be calculated [8]. In the ideal case, the exact solution of the slip line without soil weight has been proved to be a complete solution. When considering the existence of an exact solution of the slip line in soil, the current research cannot strictly prove whether it is a complete solution.

### 3.2. Thermal Analysis and Basic Theory

#### 3.2.1. Basic Theory of Heat Transfer

In a closed system, following the law of conservation of energy is equivalent to no mass inflow or outflow.

(5) $$\begin{array}{c} Q-W=\Delta U+\mathrm{\Delta KE}+\mathrm{\Delta PE}, \end{array}$$

where *Q* is heat of closed system; *W* is work done by closed system; Δ*U* is internal energy of closed system; ΔKE is kinetic energy of closed system; ΔPE is potential energy of closed system.

In many engineering heat transfer problems, the general situation is that the kinetic energy of the system is equal to the potential energy of the system and is zero; that is,

(6) $$\begin{array}{c} \mathrm{\Delta KE}=\mathrm{\Delta PE}=0. \end{array}$$

Generally, work is not considered; that is,

(7) $$\begin{array}{c} W=0,\\ Q=\Delta U. \end{array}$$

The steady-state thermal analysis and transient thermal analysis are as follows:

(8) $$\begin{array}{c} Q=\Delta U=0,\\ q=\frac{dU}{dt}. \end{array}$$

#### 3.2.2. Steady-State Analysis Theory

When the net heat flow rate of the system is 0, the system is in a thermal stable state, which can be expressed as

(9) $$\begin{array}{c} Q_{\text{input}}+Q_{\text{genreate}}-Q_{\text{output}}=0. \end{array}$$

In this state, the temperature of each node will not change with time. The equilibrium equation of thermal analysis can be expressed in matrix form:

(10) $$\begin{array}{c} \left[K\right]\left\{T\right\}=\left\{Q\right\}, \end{array}$$

where [*K*] is conduction matrix, including shape coefficient, emissivity, convection coefficient, and thermal conductivity; {*T*} is node temperature vector; [*Q*] is node heat flux vector, including heat generation [9].

### 3.3. ANSYS Analysis of Ultimate Bearing Capacity of Foundation

#### 3.3.1. Modeling and Meshing

The model built in this chapter is a cylinder with a diameter of 3 meters and a depth of 1 meter. Plane55 was used in the calculation of temperature field in the early stage, and solid70 unit was later converted to plane42 and solid45 unit in the calculation of stress field, with a total of 10669 units [10].

#### 3.3.2. Determination of Creep Parameters of Materials

The creep rate equation of generalized Kelvin model is

(11) $$\begin{array}{c} \frac{\partial \varepsilon }{\partial t}=\left(\frac{\sigma }{\eta }\right)•\exp\left(\frac{-E_{k}t}{\eta }\right). \end{array}$$

The implicit creep equation (3) provided in ANSYS is as follows:

(12) $$\begin{array}{c} \frac{\partial \varepsilon }{\partial t}=C_{1}\sigma^{C_{2}}r•\exp\left(-rt\right),\\ r=C_{5}\sigma^{C_{3}}•\exp\left(\frac{-C_{4}}{T}\right). \end{array}$$

By substitution, we have

(13) $$\begin{array}{c} \frac{\partial \varepsilon }{\partial t}=C_{1}C_{5}\exp\left(\frac{-C_{4}}{T}\right)\sigma^{C_{2}}\sigma^{C_{3}}\exp\left[-C_{5}\sigma^{C_{3}}\exp\left(\frac{-C_{4}}{T}\right)\right]. \end{array}$$

Compare equations (11) and (13) to obtain the following equation group:

(14) $$\begin{array}{c} \left\{\begin{array}{c} \frac{1}{\eta }=C_{1}C_{5}\exp\left(\frac{-C_{4}}{T}\right)\sigma^{C_{3}},\\ C_{2}=1,\\ C_{3}=0,\\ \frac{E_{k}}{\eta }=C_{5}\sigma^{C_{3}}\exp\left(\frac{-C_{4}}{T}\right). \end{array}\right. \end{array}$$

In the above equation group, *T* represents the temperature under the open temperature scale. When the test temperature is taken as 0°C, that is, *T*=273K, and the temperature is taken as 0°C, that is, *T*=258K, taking *C*_1_, *C*_2_, *C*_3_, *C*_4_, *C*_5_ as the unknowns of the equations, there are countless solutions to the equations, and the creep equations determined by any of them are equivalent [11]. Therefore, it can be taken as *C*_2_=1, *C*_3_=0, *C*_4_=5, so Table 1 can be obtained accordingly.

#### 3.3.3. Freezing Temperature Field

Thermal convection refers to the exchange of heat between the outer surface of a solid and its surrounding fluid due to the temperature difference. It occurs on the upper surface of the test model, as shown in Figure 2.

Thermal convection can be described by Newton's cooling equation.

(15) $$\begin{array}{c} q^{n}=h\left(T_{S}-T_{B}\right), \end{array}$$

where *h* is the convective heat transfer coefficient; *T*_*S*_ is the temperature of the solid surface; *T*_*B*_ is the *q*^*n*^=*h*(*T*_*S*_ − *T*_*B*_) temperature of the surrounding fluid. Heat conduction is due to the temperature difference in different parts of the interior. When the temperature is high, the heat will be transferred to the part with low temperature. This form of heat conduction occurs in the interior of the test model, as shown in Figure 3.

The formula is as follows:

(16) $$\begin{array}{c} \frac{Q}{t}=\frac{KA\left(T_{\text{hot}}-T_{\text{cold}}\right)}{d}, \end{array}$$

where *Q* is the heat transfer within time *t*; *K* is the heat conductivity coefficient; *T* is the temperature; *A* is the plane area; *d* is the distance between two planes.

#### 3.3.4. Simulated Value of Bearing Capacity

Through the data extraction of ANSYS finite element software in simulating the bearing capacity of frozen soil foundation, the displacement under different loads is obtained, and the following curve is generated, as shown in Figure 4.

Through observation and analysis of the P-S curve simulated by ANSYS software, when the foundation is frozen to −15°C stable state, after staged loading, from the analysis of the diagram, when the load is about 190 kN, the trend of the curve changes significantly [12]. The bearing capacity in the P-S curve measured in the indoor similar model test is 170 kN. There is a difference between the two, but the difference is not too great. Because ANSYS software simulates the foundation bearing capacity under ideal conditions, there will be some deviation between the measured value and the simulated value.

## 4. Field Bearing Capacity Model Test of Special Water Conservancy Foundation

### 4.1. Project Overview and Selection of Test Area

The test site is reclaimed from the sea, backfilled with mountain broken stone soil, and treated by dynamic compaction. The terrain is relatively flat, low in the South, and high in the north, which has better drainage advantages. According to the detailed geotechnical investigation technical report, there are six genetic types of strata within the maximum exposed depth of 42.1 m in the investigation site. The test area is selected in the area where the muddy silty clay layer is thick and there is no important structure on the upper part. In combination with the geological exploration report and the site layout plan, the pilot area is preliminarily selected to be located near zk932, z1092, and zk931 boreholes. The three exploration holes reveal that the thickness of the sludge layer is about 10 m and the filling layer is about 4–6 m. Three test areas are arranged in this test, and three test piers are arranged in each test area. The three test piers in test area 1 are 1-1, 1-2, and 1-3; the three test piers in test area 2 are 2-1, 2-2 and 2-3; The three test piers in test area 3 are 3-1, 3-2 and 3-3 [13]. See Table 2 for test pier parameters.

The foundation reinforcement treatment in the three test areas is divided into two construction processes: preformed hole deep compaction bag gravel pier method and preformed hole deep compaction bag gravel pier method [14]. These two methods are used to reinforce the foundation of three test areas. There are three test piers in each test area. Two pier bodies are selected for preformed hole deep compaction bag gravel pier method, and one pier body is selected for preformed hole deep vibration bag gravel pier method, and then gravity penetration test is used to detect the compactness of pier body. See Table 3 for the construction process of 9 pier bodies in three test areas.

The main machines and tools for this test construction are shown in Table 4.

The construction technology of this test is preformed hole deep compaction bag gravel pier method. A total of six pier bodies were selected in the three selected test areas for predrilled deep compacted bag pier foundation treatment [15]. The construction site conditions in this test area can meet the requirements of mechanical equipment walking and running in the site, and various construction machines and tools can smoothly enter the construction site for testing. There are 9 test piers of bag gravel pier, which are divided into 3 groups. The first group is the test of 1-1, 1-2 and 1-3 gravel piers. The hole diameter is 800 mm, and there is no geotextile bag. The second group is the test of 2-1, 2-2, and 2-3 gravel piers, with a hole diameter of 800 mm and geotextile bags. The third group is 3-1, 3-2, and 3-3 gravel piers, with a hole diameter of 1200 mm and geotextile bags. See Table 5 for details.

The calculation method of test filling coefficient is as follows:

(17) $$\begin{array}{c} Filling\;factor=\frac{Actual\;filling\;amount}{Actual\;pile\;length\times Drilling\;radius^{2}\times \pi }. \end{array}$$

It can be seen from Table 5 that the filling coefficient of test area 1 is significantly greater than that of test areas 2 and 3; that is, the filling coefficient of gravel pier without geotextile bag is significantly different from that of gravel pier with geotextile bag. The filling coefficient of gravel pier without geotextile bag is larger than that of gravel pier with geotextile bag. If the filling coefficient is too large, it indicates that the actual pouring amount is less than the theoretical calculation amount, and the quality of the pier body has defects. If the filling coefficient is too large, it indicates that the geological conditions of the test site are poor, and the filler of the pier body diffuses and compresses to the surrounding soil. Comparing test areas 1 and 2, it can be found that, in test area 2, the filling coefficient decreases after the pier is wrapped with geotextile bags, indicating that the pier wrapped with geotextile bags can effectively limit the diffusion of pier filler and control the filling coefficient of pier within a reasonable range.

### 4.2. Ultraheavy Dynamic Penetration Test

#### 4.2.1. Test Method

The test's purpose is as follows: super heavy dynamic penetration test is used to detect the compactness of gravel pier body; YZ-100 drilling rig is adopted as the drilling equipment; the falling weight is 120 kg and the falling distance is 100 cm.

1. Before penetration, install the sounding frame steadily to keep the sounding hole vertical, and the maximum deflection shall not be greater than 2%.
2. During the test, the falling hammer falls freely and penetrates continuously, and the hammering rate is 15∼30 blows/min.
3. Record the number of blows required for each 10 cm of penetration.
4. Rotate the probe rod for one and a half circles every 1 m of penetration; when the penetration depth exceeds 10 m, rotate the probe rod once every 20 cm.
5. Process data, draw the relationship curve between the number of blows (N120) and the penetration depth (*H*), analyze the test data, and evaluate the foundation treatment effect [16].

#### 4.2.2. Test Results and Analysis

According to the analysis of the test process and test results, the test process is mainly controlled from the pier shaft diameter, whether to set bags, vibration retention time, filler amount, filler particle gradation, and other parameters. The parameters and test results are shown in Table 6.

It can be seen from Table 6 that test area 1 is the gravel pier without geotextile bags, with an average number of dynamic detection blows of 3.87, test area 2 is the gravel pier with geotextile bags, with an average number of dynamic detection blows of 5.57, test area 3 is the gravel pier with geotextile bags, with an average number of dynamic detection blows of 4.27, and the average number of dynamic detection blows of test areas 2 and 3 is 4.92, which is significantly greater than that of test area 1. It is shown that geotextile bags have an obvious effect on improving the compaction effect of pier body. Super heavy dynamic penetration test was carried out in three test areas, and two pier forming methods were tested. It can be seen from Table 6 that test area 1 is the gravel pier without geotextile bags, with an average number of dynamic detection blows of 3.87, test area 2 is the gravel pier with geotextile bags, with an average number of dynamic detection blows of 5.57, test area 3 is the gravel pier with geotextile bags, with an average number of dynamic detection blows of 4.27, and the average number of dynamic detection blows of test areas 2 and 3 is 4.92, which is significantly greater than that of test area 1. It is shown that geotextile bags have an obvious effect on improving the compaction effect of pier body. Super heavy dynamic penetration test was carried out in three test areas, and two pier forming methods were tested. Draw the relationship curve between the number of blows (N120) and the penetration depth (*H*), analyze the test data, and evaluate the foundation treatment effect [17]. The relationship curve between blow counts (N120) and penetration depth (*H*) in the three test areas is shown in Figure 5.

It can be seen from Figure 5 that, within 3 meters of the top, the pier 1-1 body is hit 3 times, the pier 1-2 body is hit 2 times, and the pier 1-3body is hit 2 times; that is, the pier body within 3 meters of the top of the pier body is in a loose state, which is not conducive to bearing the upper load. For the three pier bodies in the test area, the number of blows of pier 1-3bodies is greater than those of pier 1-1 bodies and pier 1-2 bodies, indicating that the compactness of the vibrated bag gravel pier method in test area 1 is greater than that of the compacted bag gravel pier method. The average number of blows of the three test piers in test area 1 is 3.9, and the compactness of the pier body is slightly dense [18]. The relation curve between load (P) and settlement (S) of piers 1-3, 2-3, and 3-3 before full compaction reinforcement is shown in Figure 6.

According to the P∼S curve and test data, the settlement of pier 1-3 exceeds 4 cm after being loaded to 540 kN, and the curve is slowly changing. Taking the total settlement S of the pile top as 40 mm, the corresponding load value of 495 kN is the limit value of the vertical compressive bearing capacity of a single pile, so the characteristic value of the vertical compressive bearing capacity of a single pier 1-3 is 247.5 kN.

The settlement of pier 2-3 exceeds 4 cm after being loaded to 810 kN, and the curve shows a gradual change. Taking the total settlement S of the pile top as 40 mm, the corresponding load value 725 kN is the limit value of the vertical compressive bearing capacity of a single pile, so the characteristic value of the vertical compressive bearing capacity of a single pier 2-3is 362.5 kN.

The settlement of pier 3-3 exceeds 4 cm after being loaded to 1260 kN, and the curve is slowly changing. Taking the total settlement of pile top S as 40 mm, the corresponding load value 1177 kN is the limit value of vertical compressive bearing capacity of single pile, so the characteristic value of vertical compressive bearing capacity of single pile of test pile in zone 3 is 588.5 kN. See Table 7 for the summary of test results.

It can be seen from Figure 6 that the P∼S curve in the test area has no obvious proportional limit, which is a slowly varying curve. Within the range of ultimate bearing capacity of test area 1, under the same load, the settlement of test area 1 is always greater than that of test areas 2 and 3, indicating that geotextile bags provide lateral constraints for the pier body to limit lateral deformation, improve the bearing capacity of the pier body, and reduce the foundation settlement [19]. In comparison between test areas 1 and 2, when *p* < 400 kPa, the average settlement of test area 1 is 12 mm larger than that of test area 2 under the same load. When *p* > 400 kPa, the settlement difference increases significantly with the increase of load P, indicating that, under the load, the lateral restraint provided by geotextile bags improves the compressive bearing capacity of piers, and, with the increase of load, the role of geotextile bags in limiting the lateral extrusion of gravel particles is more significant. In comparison between test areas 2 and 3, when *p* < 300 kPa, the P∼S curves of test zone 2 and test zone 3 are basically similar. When *p* > 300 kPa, under the same load, the settlement of test zone 3 is greater than that of test zone 2, and, with the increase of load P, the settlement difference increases significantly, indicating that the larger the pier diameter of geotextile bag gravel pier is, the greater the compressive capacity of pier body is and, with the increase of load, the greater the pier diameter to the compressive capacity of pier body is. In comparison between test areas 1 and 3, the bearing capacity of pier 3-3 is about twice that of pier 1-3, but the settlement is not much different, indicating that geotextile bags can improve the bearing capacity of pier body, limit the deformation of pier body, and reduce the settlement. Through the analysis of the results of the super heavy dynamic penetration test, it can be seen that the upper part of the pile is in a loose state within about 3 M, and the static load test cannot accurately show the vertical bearing capacity of the pier body due to its influence. Therefore, the pier body was fully compacted, and the static load test was carried out on the pier body after full compaction. The relationship curve between load (P), kPa, and settlement (S), mm, is shown in Figure 7, and the summary of the test results is shown in Table 8.

It can be seen from Figure 7 that, under the same load, the settlement after full compaction is significantly reduced compared with that before compaction. When test area 3 is loaded to 3600 kN, there is still no steep drop section in the P∼S curve. Taking the total settlement S of the pile top as 40 mm and the corresponding load value of 2955 kN as the limit value of the vertical compressive bearing capacity of the single pier, the characteristic value of the vertical compressive bearing capacity of the single pier is 1477 kN, about 2.5 times that before reinforcement [20]. It is shown that the compactness of the pier body within the depth range of 2∼3*D* (*D* is the pier diameter) of the geotextile bag gravel pier has a significant impact on the vertical bearing capacity of the single pier. The higher the compactness is, the greater the vertical bearing capacity of the single pier is.

### 4.3. Model Test Results of Artificial Frozen Soil under Load

The purpose of this model test is to test the structural response of seasonally frozen soil foundation under cyclic load and the corresponding frozen soil foundation parameters, to determine the failure mode of frozen soil foundation under reciprocating load and the characteristics of its load transmission and to analyze the influence of temperature on the bearing capacity, so as to provide support for theoretical analysis and numerical calculation. The following equipment is used in this test: large multifunctional artificial freezing platform, temperature sensor (thermocouple), displacement sensor, load sensor, ye2532 static strain collector, oil pump, oil jack, computer, and so forth [21]. The platform used in this test has a diameter of 3.0 m and a depth of 0.9 m. The test platform is filled with clay as the test soil. Clay is filled and compacted in layers. The artificial freezing method is used in the soil refrigeration process, and the refrigeration liquid (cooled alcohol) will reach each circle of circulating pipes from the main inlet and return pipelines. After that, the liquor semen circulation tube enters the vertical freezing tube wrapped with a protective layer. The lower end of the vertical freezing pipe in the depth drawing is sealed. The outer diameter of the freezing pipe is 20 mm and the inner diameter is 14 mm. The cooled alcohol enters from the liquid inlet pipe, flows into the freezing pipe, and then flows out from the liquid return pipe. In this way, the heat in the soil can be dissipated, so that the soil in the pit is cooled and frozen. Each freezing pipe is not imaginative and will not be affected by adjacent pipes, so as to ensure that the soil freezing effect is relatively uniform [22].

#### 4.3.1. Bearing Capacity Test of Frozen Soil Foundation

In this test, considering that the strength and deformation of foundation soil will be affected by temperature changes, the static load test method is used to test frozen soil foundation. The fill is Huainan local soil, and its physical property indexes are shown in Tables 9 and 10, which show the deformation modulus and Poisson's ratio of frozen soil, thawed soil, and normal temperature soil.

First measure the initial moisture content of the soil, calculate the amount of water needed according to the preset moisture content, sprinkle water, turn over and mix, and prepare a large number of soils required for the test for use [23].

#### 4.3.2. Test Method

The ye2532 static strain gauge mentioned above was used for all data collection of the test, as shown in Table 11.

According to the regulations and requirements on shallow plate load test, this test adopts the method of applying load by stages on the rigid bearing plate with a diameter of 300 mm by using the jack, adopts the rapid maintenance load method, adds a level of load every 1 H, tests the settlement of frozen soil under all levels of load, and obtains the load settlement (P-S) curve under all levels of load [24]. Among them, the loading stage is set as 8 levels; that is, loading is carried out in eight times, and the load of each level gradually increases. The load of the first level is about 15%–30% of the preestimated limit load, and then the load applied each time should be 10%–15% of the estimated load.

#### 4.3.3. Test Results and Analysis

The P-S results are given in Table 12.

According to the previous theoretical summary, when there is a clear proportional limit on the P-S curve, the proportional limit can be taken as the load value. When the limit load value is less than 2 times of the corresponding proportional limit load value, take half of the limit load value as the load value. The above two values can take the lowest value. According to the observation and analysis in Figure 8, when the foundation temperature is kept at −15°C, the proportional limit points on the two P-S curves are the same, and the load shows 170 kN. 170 kN is taken as the foundation bearing capacity of the circular area with a diameter of 300 mm, that is, 2.41 MPa. The temperature decreased from 0°C to −15°C, and the bearing capacity of the foundation increased by more than 20 times. This is mainly because the temperature drops below 0°C, and the pore water of the foundation soil is transformed into pore ice, resulting in changes in the internal structural connection in the soil. The pore ice firmly binds the mineral particles in the soil together, which greatly enhances the mechanical indexes of the foundation, and the bearing capacity of the foundation is greatly improved. The determination of foundation bearing capacity is crucial in the design of foundation. Therefore, the determination of foundation bearing capacity of frozen soil under freezing conditions through tests is also critical for application in practical projects [25–34]. Through the test and analysis in this chapter, it is concluded that when the temperature gradually decreases, due to the cementation of ice in the soil, the bearing capacity of the foundation will significantly increase. For the determination of the bearing capacity of frozen soil foundation, there are many impression factors. Freezing temperature, physical and mechanical properties of soil, foundation width, buried depth, and other factors affect the bearing capacity of frozen soil foundation.

## 5. Conclusion

In this paper, the compressive strength test and uniaxial creep characteristic test of frozen soil foundation are carried out. The physical and mechanical properties of artificially remolded soil are measured under the conditions of −5°C, −10°C, and −15°C freezing temperature and water content of 20%, 25%, and 30%, respectively. Through indoor model test, static load test method and finite element software simulation method are used to analyze the bearing capacity of frozen soil foundation, and the main conclusions of this paper are listed as follows:

1. Due to the difference of freezing temperature, the compressive strength of artificially frozen clay foundation increases gradually with the decrease of temperature, which is close to linear growth.
2. The compressive strength of frozen soil foundation is affected by the difference of water content. When the temperature is getting lower and lower, the influence will become more and more obvious. The uniaxial creep attenuation curve of artificial frozen soil is relatively scattered. When the loading coefficient is set to be large, the creep development of the sample will have an obvious different trend due to the different freezing temperature.
3. The finite element software ANSYS can effectively simulate complex boundary conditions and initial conditions, first use the temperature field theory to reach the corresponding temperature of the foundation soil, form a steady-state temperature field, and then apply load to the frozen soil foundation to simulate the whole stress field.
4. In ANSYS, the incremental load method is used to solve the ultimate bearing capacity, which is convenient to operate. Through simulation, the response curve of the load to the foundation can be obtained, the load value with relatively high accuracy can be obtained, and the destruction of frozen soil foundation can be visualized, which provides a foundation for the analysis of practical projects in the future.

## Figures and Tables

**Figure 1:** Bearing capacity model of water conservancy land foundation.

**Figure 2:** Convection diagram.

**Figure 3:** Heat conduction diagram.

**Figure 4:** P-S diagram.

**Figure 5:** N120∼H curve of ultraheavy dynamic penetration test in test area 1 (800 mm without geotextile bag).

**Figure 6:** P∼S curve of plate load test before full compaction and reinforcement.

**Figure 7:** P∼S curve of plate load test after full compaction and reinforcement.

**Figure 8:** Load settlement (P-S) curve of frozen soil foundation.

**Table 1:** Creep parameters.

	Loading factor	*η*	*E*_*k*_	*C*_1_	*C*_2_	*C*_3_	*C*_4_	*C*_5_
0°C	0.3	0.043	0.03866	26.53	1	0	5	0.8523
	0.5	0.01788	0.02427	41.187	1	0	5	1.3866
	0.7	0.00856	0.03319	30.142	1	0	5	3.945

−15°C	0.3	1.0243	1.3839	0.723	1	0	5	1.378
	0.5	1.1673	2.3	0.436	1	0	5	2.0036
	0.7	0.13	0.138	7.198	1	0	5	1.181

**Table 2:** Test parameters.

Test area	Hole diameter (mm)	Bag diameter (mm)	Quantity	Pier length (m)	Bag strength
Test area I	800	No cloth bag	3	13	HP470
Test area II	800	1000	3	13	HP470
Test area III	1200	1400	3	13	HP470

**Table 3:** Construction process of three test areas.

Test area	Pier number	Construction technology
Test area I	1-1	Tamping bag gravel pier method
	1-2	Tamping bag gravel pier method
	1-3	Vibrating bag gravel pier method

Test area II	2-1	Tamping bag gravel pier method
	2-2	Tamping bag gravel pier method
	2-3	Vibrating bag gravel pier method

Test area III	3-1	Tamping bag gravel pier method
	3-2	Tamping bag gravel pier method
	3-3	Vibrating bag gravel pier method

**Table 4:** Main machines and tools.

Serial number	Name	Specification and model	Rated power (kW) or tonnage (*t*)	Quantity
1	Dynamic compaction machine	400-AF	—	1
2	Rotary drilling rig	FR620C	195 kW	1
3	Hydraulic vibratory hammer	ICE416L	262 kW	1
4	Loader	ZL50C	13 kW	2
5	Total station	Topcon102N	—	1
6	Measuring rope	50 m	—	1
7	Steel rule	5 m	—	1
8	Vibrating rod	12.5 m	—	2

**Table 5:** Statistics of construction process parameters and results.

Number	Hole diameter (mm)	Bag diameter (mm)	Pier length (m)	Cloth bag	Total filler volume (m^3^)	Filling coefficient	Filling times	Vibration retention time (min)	Vibration retention times	Filler particle size (mm)
1-1	800	900	13.5	Nothing	13.0	1.37	7	Tamp	—	5–10
1-2	800	900	14	Nothing	14.1	1.45	7	Tamp	—	5–10
1-3	800	900	13	Nothing	13.1	1.45	8	31.4	8	5–10
2-1	800	900	13	Have	12.7	1.10	7	Tamp	—	5–10
2-2	800	900	13	Have	11.1	1.23	8	Tamp	—	5–10
2-3	800	900	13	Have	12.3	1.16	7	35	7	5–10
3-1	1200	1200	14	Have	16.1	1.33	8	Tamp	—	5–10
3-2	1200	1200	13	Have	14.7	1.10	8	Tamp	—	5–30
3-3	1200	1200	13	Have	14.8	1.13	7	37.4	7	5–30

**Table 6:** Statistical table of dynamic penetration test results.

Number	Hole diameter (mm)	Cloth bag	Total filler volume (m^3^)	Vibration retention time (min)	Average dynamic detection hits (*n*)	Estimation of characteristic value of bearing capacity of single pier (kN)
1-1	800	Nothing	13.0	Tamp	2.9	148.98
1-2	800	Nothing	14.1	Tamp	3.1	159.4
1-3	800	Nothing	13.1	31.4	5.3	247.3
2-1	800	Have	12.7	Tamp	5.1	221.1
2-2	800	Have	11.1	Tamp	5.0	210.2
2-3	800	Have	12.3	35	6.3	358.6
3-1	1200	Have	16.1	Tamp	3.2	367.8
3-2	1200	Have	14.7	Tamp	3.8	401.3
3-3	1200	Have	14.8	37.4	5.3	584.7

**Table 7:** Vertical compressive static load test results of single pier.

Test pier no.	Pier length (m)	Pier diameter (mm)	Area of pressure bearing plate (m^2^)	Ultimate bearing capacity (kN)	Maximum settlement (mm)	Characteristic value of bearing capacity (kN)	Corresponding settlement (mm)
1-3	13	1000	0.63	494	45.00	247.4	15.76
2-3	13	1000	0.63	724	40.00	361.4	14.96
3-3	13	1200	0.94	1176	46.00	588.4	15.85

**Table 8:** Vertical compressive static load test results of single pier.

Test pier no.	Pier length (m)	Pier diameter (mm)	Area of pressure bearing plate (m^2^)	Ultimate bearing capacity (kN)	Maximum settlement (mm)	Characteristic value of bearing capacity (kN)	Corresponding settlement (mm)
1-3	13	1000	0.63	1350	32.00	674	19.76
2-3	13	1000	0.63	2250	30.00	1124	16.94
3-3	13	1200	0.94	2955	40.00	1476	18.85

**Table 9:** Physical property index of fill.

Soil sample	Moisture content (%)	Density (g/cm^3^)	Porosity (%)	Liquid limit (%)	Saturation (%)	Plastic limit (%)
Normal temperature clay	23.1	1.789	0.706	35.6	1.00	19.2
Frozen soil		1.720				
Thawed soil	24.5	1.7	0.71	33.2	1.01	19.06

**Table 10:** Deformation modulus and Poisson's ratio of frozen soil, thawed soil, and normal temperature soil.

	Conventional soil	Thawed soil	Frozen soil		
			−5°C	−10°C	−15°C
Elastic modulus *E*/MPa	2.6	0.25	62.8	110.3	191.6
Poisson's ratio *μ*	0.34	0.34	0.22	0.21	0.17
Cohesion C/kPa	7.21	4.31	137	191	240

**Table 11:** Test load values at all levels.

Classification serial number		1	2	3	4	5	6	7	8
Load value (kN)	*T* = 0°C	3.6	5.1	6.4	8.1	9.6	11.1	12.6	14.1
	*T* = −15°C	80	110	140	170	200	230	260	290

**Table 12:** Load settlement of frozen soil foundation (P-S test results).

Classification serial number			1	2	3	4	5	6	7	8
*T* = 0°C	Load value (kN)		3.3	5.0	6.3	8.0	9.3	11.0	12.3	14.0
	Settlement (mm)	Measuring point 1	2.3	3.1	4.1	6.1	8.1	11.5	16.1	30.1
		Measuring point 2	2.1	3.1	4.0	5.3	7.1	10.1	16.1	28.4

*T* = −15°C	Load value (kN)		80	110	140	170	200	230	260	290
	Settlement (mm)	Measuring point 1	2.2	3.6	5.4	7.1	10.3	14.2	19.6	28.3
		Measuring point 2	2.5	4.1	5.5	7.4	10.6	15.2	20.2	29.5

## Data Availability

The dataset can be accessed upon request.
